The article "Preparation and Performance Analysis of Bacterial Cellulose-Based Composite Hydrogel Based on Scanning Electron Microscope" was retracted in 2023. Reasons: unreliable results or conclusions; concerns about the data; concerns about the peer review; concerns about the citations.

# Preparation and Performance Analysis of Bacterial Cellulose-Based Composite Hydrogel Based on Scanning Electron Microscope

**DOI:** 10.1155/2022/8750394

**Published:** 2022-08-06

**Authors:** Meiling Shao, Zhan Shi, Bin Zhai, Xiangfei Zhang, Zhongyi Li

**Affiliations:** College of Chemistry and Chemical Engineering, Shangqiu Normal University, Shangqiu, Henan 476000, China

## Abstract

In order to better prepare and analyze bacterial cellulose-based composite hydrogels, an experimental method based on scanning electron microscopy was proposed. The specific content of the method is to observe the hydrogel through scanning electron microscope, to observe the space between molecules through experiments, and to improve the effect of bacterial cellulose preparation of hydrogel. The experimental results show that the gel preparation effect is best when PEG concentration is not more than observed by scanning electron microscope. It is better to prepare bacterial cellulose complex hydrogel by scanning electron microscopy.

## 1. Introduction

Scanning electron microscope (SEM) is a kind of observation means between transmission electron microscope and optical microscope [1]. It uses a very narrow focused high-energy electron beam to scan the sample. Through the interaction between the beam and the material, various physical information is stimulated, and the information is collected, amplified, and reimaged to achieve the purpose of characterization of the microscopic morphology of the material. New scanning electron microscopes have a resolution of 1 nm. Magnification can reach 300,000 times and above continuous adjustable. In addition, scanning electron microscope and other analysis instruments can be combined to observe the microscopic morphology and analyze the composition of the material in small areas. Scanning electron microscope is widely used in the study of rock and soil graphite ceramics and nanomaterials. Therefore, scanning electron microscope plays an important role in scientific research.

The signals used for scanning electron microscopy imaging come from the interaction of the incident light beam with atoms at different depths in the sample. Under electron beam bombardment, the samples will produce many kinds of signals including back scattering, electron secondary electron, characteristic X-ray, absorption electron, transmission electron, auger electron, cathode fluorescence electron, and beam induced effect [2–4]. While it is difficult for a single machine to have all the detectors, the backscattered electron (BSE) and secondary electron (SEI) characteristic X-ray detector is the standard detector of general scanning electron microscopes.

The article "Preparation and Performance Analysis of Bacterial Cellulose-Based Composite Hydrogel Based on Scanning Electron Microscope" was retracted in 2023. Reasons: unreliable results or conclusions; concerns about the data; concerns about the peer review; concerns about the citations.

Cellulose is the most abundant natural biodegradable polymer in the world, which exists widely in the plant kingdom and is one of the main research objects in the birth and development stage of polymer chemistry [5].  Figure 1 shows the preparation of the collagen-based hydrogels. At present, there are two kinds of different ways to obtain cellulose. One is natural synthetic cellulose, which is synthesized by plants through photosynthesis or by microorganisms. The other is synthetic cellulose, which is synthesized by enzyme-catalyzed synthesis of cellulose and glucose from ring-opening polymerization of neopentyl derivatives in vitro. Synthetic cellulose has lower crystallinity and less regular morphology than natural cellulose. In today's world facing four major problems of population, resources, environment, and food, renewable natural resources have important strategic significance for sustainable development [6, 7].

In addition to plant cellulose, microorganisms can also ferment to produce cellulose, which is collectively known as bacterial cellulose [8]. When using Acetobacter xylantoides for static culture, Pfdab et al. found that a membrane formed on the surface of the medium, which was named BC after physical and chemical analysis, confirmed that it had a structure similar to cellulose [9]. According to the research, bacterial cellulose is a chain polymer composed of glucopyranose residue to residue to glycosidic bond *β* − 1. It has nanometer ultrafine network structure and has more excellent characteristics than natural plant cellulose, such as high purity, high crystallinity, large specific surface area, good hydrophilicity and biocompatibility, and easy to degrade in the environment. At present, in developed countries, bacterial cellulose industry has initially formed an annual value of more than 100 million dollars of market, involving food, chemical, pharmaceutical, textile, and papermaking industries. As a kind of environmentally friendly and renewable biological material, bacterial cellulose has great commercial value and good development prospect under the situation of increasing population and resource shortage in the world.

## 2. Literature Review

Bacterial cellulose exists in the form of pure cellulose and has a similar structure to cellulose produced by plants or algae, with unique physical and chemical properties. BC has a dense three-dimensional network structure, and the fiber diameter is between 30 and 100 nm, which is 1/10-1/100 of the plant cellulose fiber. The bacteria that can produce cellulose are mainly acetic acid bacteria, rhizobia, soil bacteria, octadiococcus, etc. The most effective species used in microbial research is the Gram-negative Acetobacter xylinoides, which was renamed as Gluconacetobacter xylinus internationally.

The article "Preparation and Performance Analysis of Bacterial Cellulose-Based Composite Hydrogel Based on Scanning Electron Microscope" was retracted in 2023. Reasons: unreliable results or conclusions; concerns about the data; concerns about the peer review; concerns about the citations.

Studies on bacterial cellulose synthesis contribute to a better understanding of the biological origin of plant cellulose. At the beginning, the research on BC biosynthesis has been limited to physiological and biochemical properties, but in recent decades, with the development of molecular biology, the research on the mechanism of BC biosynthesis has been accelerated. The synthesis of bacterial cellulose is a specifically controlled multistep reaction process involving a complex system of unique enzymes that catalyze and regulate protein reactions. These processes include the synthesis of the cellulose precursor glucose uridine diphosphate, followed by glucose polymerization *β* − 1, and the synthesis of 4-glucan chains, whereby the terminal complex continuously transfers pyranoid glucose residues from UDPGlu to the newly formed polysaccharide chain. Supramolecular network structure was thus formed. The synthesis pathway of UDPGlu has been reported, but the molecular mechanism of the assembly and combination of multiple dextran chains into fibrils needs to be further elucidated.

The pentose phosphate cycle and tricarboxylic acid cycle are two main metabolic pathways in cellulose synthesis by Acetobacter xylantoides. The pentose phosphate cycle is a metabolic process through glucose alienation and effective sugar alienation synthesis of cellulose. Because of the possibility of mutual conversion between pyruvate and glucose, the glycolysis pathway should be inhibited so that pyruvate is continuously converted to glucose. In the tricarboxylic acid cycle, glycogen dissimilation occurs from oxaloacetate through pyruvate, oxaloacetate declothase, and pyruvate kinase, and hexose phosphate synthesizes cellulose through isomerization and phosphorylation. When the energy charge is high, that is, when the activity of 6-phosphate glucose dehydrogenase is inhibited by ATP, glucose metabolism is conducive to the synthesis of cellulose, whereas glucose metabolism enters HMP (Table 1).

In view of this research problem, Ji et al. believed that bacterial cellulose in wet state had high tensile strength, high elastic modulus, high water holding capacity, and smooth internal and external surface, which could be used as artificial blood vessels in surgery [10]. Vasava and Panchal believed that bacterial cellulose had a special three-dimensional network structure, high wet strength, high water absorption, and water retention due to nanoeffect and could be formed by in situ processing in wet state. Because of its high purity and excellent performance, bacterial cellulose fiber can be widely used in medical dressings, tissue engineering scaffolds, artificial blood vessels, artificial skin, and other aspects. It is one of the hot fields of international biomedical material research [11]. Babu believes that the combination of scanning electron microscope and other analytical instruments can be used to observe the microscopic morphology and analyze the composition of the material in small areas [12].

The article "Preparation and Performance Analysis of Bacterial Cellulose-Based Composite Hydrogel Based on Scanning Electron Microscope" was retracted in 2023. Reasons: unreliable results or conclusions; concerns about the data; concerns about the peer review; concerns about the citations.

An experimental method based on scanning electron microscope is proposed in this paper. The specific content of this method is to observe the hydrogel through scanning electron microscope and observe the intermolecular space through experiment to prove the effect of this method to solve the problem of preparing hydrogel from bacterial cellulose.

## 3. Method

### 3.1. Secondary Electron Morphology Contrast Principle

Secondary electron is a kind of free electron produced by bombarding the sample with an electron beam so that the outer electrons of the atom in the sample are separated from the atom. Secondary electron has a lower energy, generally less than 50 eV. Since the secondary electrons are generated very close to the surface of the sample (generally 5-10 nm away from the surface), the secondary electron imaging (SEI) can characterize the sample surface with a high resolution up to 1 nm.

### 3.2. Principle of Atomic Number Contrast of Backscattered Electrons

Backscattered electrons (BSE) are part of the electrons reflected by the sample in the process of electron beam bombardment, including elastic backscattered electrons reflected by the nucleus and inelastic backscattered electrons reflected by the outer nucleus. The scattering angle of elastic backscattering electrons is greater than 90, and there is no energy loss. Therefore, the energy of elastic backscattering electrons is very high, generally reaching thousands to tens of thousands of volts. Inelastic backscattering electrons not only change direction but also have different degrees of energy loss due to collision with exonuclear electrons. Therefore, the energy distribution range of inelastic backscattering electrons is wide, generally tens of electron volts to thousands of electron volts. Since inelastic backscattered electrons need to be scattered many times before escaping from the sample surface, the number of inelastic backscattered electrons is much higher than that of inelastic backscattered electrons. Therefore, the backscattered electrons referred to in scanning electron microscopy mostly refer to elastic backscattered electrons. The resolution of the backscattered electron image is lower than that of the secondary electron image because the backscattered electron image is generated at a depth of several hundred nanometers from the sample surface. However, the yield of backscattered electrons is highly dependent on the atomic number of the sample, so it can be used to provide information on the atomic number contrast of the sample. In the backscattering mode, the region with large average atomic number on the sample surface has strong backscattering signal, which shows high brightness in the electron microscope image. On the contrary, the region with small atomic number is dark. Therefore, in the analysis of scanning electron microscope, backscattered electrons are usually combined with the energy spectrum produced by characteristic X-ray to do composition analysis. In addition, because the intensity of backscattered signal is related to the angle between the sample crystal plane and the incident electron beam, when the angle between the incident electron beam and the crystal plane is larger, the backscattered signal is stronger, and the image is brighter and vice versa; the backscattered electron can be used for crystal orientation analysis [13, 14].

The article "Preparation and Performance Analysis of Bacterial Cellulose-Based Composite Hydrogel Based on Scanning Electron Microscope" was retracted in 2023. Reasons: unreliable results or conclusions; concerns about the data; concerns about the peer review; concerns about the citations.

### 3.3. Principle of Characteristic X-Ray and Application of Energy Spectrum

When the high-energy electron beam bombards the sample and ionizes the electrons in the inner layer of the atom in the sample, the atom at this time is in a high excited state, and the high-energy electrons in the outer layer will transition to the inner layer to fill the vacancy in the inner layer and release energy, which is called characteristic X-ray. These characteristic X-rays can be used to identify components and determine the abundance of elements in samples.

### 3.4. Experiment Reagent

Experimental reagents and instruments are shown in Tables 2 and 3.

### 3.5. Minimal Medium

1. Inclined surface medium for Acetobacter xylantoides: glucose 25 g/L, peptone 3 g/L, yeast extract 5 g/L, agar sterilization 18 g/L, and pH 5; the sterilization was conducted under 121°C for 20 min (3 strains all use the same inclined plane medium)
2. Seed solution of Acetobacter xylantoides slant medium
3. Glucose 25 g/L, peptone 3 g/L, yeast extract 5 g/L, and pH 5.0; the sterilization was conducted under 121°C for 20 min
4. Fermentation medium for Acetobacter xylantoides seed liquor
5. Fermentation medium: carbon source 25 g/L, peptone 3 g/L, and yeast extract 5 g/L; the sterilization was conducted under 121°C for 20 min
6. Note: the carbon source is xylose glucose, arabinose galactose, or mannose

#### 3.5.1. Acetobacter xylostella Seed Rejuvenation

The medium used for rejuvenation is liquid seed medium, and the configuration method is shown in 3.4 [15]. The seed medium and activated strain inclined surface were taken, and two ring strains were selected by inoculation ring and inserted into 100 mL liquid medium. The whole process was sterile operation. After the medium was shaken well, it was placed in a temperature-controlled shaker and incubated at a speed of 160 RPM for 24 hours.

The article "Preparation and Performance Analysis of Bacterial Cellulose-Based Composite Hydrogel Based on Scanning Electron Microscope" was retracted in 2023. Reasons: unreliable results or conclusions; concerns about the data; concerns about the peer review; concerns about the citations.

#### 3.5.2. Preparation of Bacterial Cellulose Membrane

The finished seed liquid was inoculated into 100 mL different fermentation medium by 6% (vt%) and incubated for 30 days at constant temperature. Gel-like bacterial cellulose film with certain thickness was generated at the interface between medium and air [16].

#### 3.5.3. Posttreatment of Bacterial Cellulose Membrane

The bacterial cellulose membrane, which had been incubated for 10 days, was removed and rinsed with deionized water. After 2 hours immersion in NaOH aqueous solution of 0.1% (wt%) at 80 °C, they were then immersed in deionized water at 80 degrees Celsius for two hours. Cyclic treatment was performed at least 3 times to remove the remaining thallus and culture medium, resulting in a transparent gel-like bacterial cellulose membrane. Rinse repeatedly with deionized water until the pH is about 7, and the film appears milky and translucent [17]. Put it into deionized water and store it at room temperature after sterilization for 20 min. The wet film is bacterial cellulose. The wet film is quick-frozen with liquid nitrogen and then freeze-dried with a freeze dryer to obtain bacterial cellulose dry [18].

#### 3.5.4. Effects of Inoculum Amount on Bacterial Cellulose Yield and Fermentation Initiation on Bacterial Cellulose Yield

Three strains of Acetobacillus xyloides used fermentation medium of E -carbon source D-grapes.The shaking time of the seed solution was 30 hours.Then the inoculum was inoculated into 50ml of fermentation medium at 2%, 4%, 6%, 8% and 10%. The initial pH was 5.5 and incubated at 30°C for 10 days. The initial pH was 5.5 and incubated at 30°C for 10 days.Bacterial cellulose membranes were harvested and then dried, weighed and averaged.

The fermentation medium of three strains of A. xylobacter strains is D-glucose. The shaking time of seed liquid was then inoculated into fermentation medium according to the inoculation amount, starting at 4, 4.5, 5, 5.5, and 6. The bacterial cellulose film was harvested and then dried and weighed for average value [19].

Orthogonal experiment design is to use mathematical statistics and orthogonality principle, through the reasonable arrangement of experiments, through a few test times, quickly obtain experimental results [20]. Orthogonal experiment is within the scope of the investigation; the purpose of the selected typical minority test conditions and find the best condition of production and scientific research Selecting strains of ages and the quantity of the experiment, to design the orthogonal scheme with three factors three levels, each child three parallel experiment, initial 5, fermentation time for 10 days, harvest bacterial cellulose membrane Then dry weight average.  Table 4 shows the orthogonal experimental factors and level tables.

The article "Preparation and Performance Analysis of Bacterial Cellulose-Based Composite Hydrogel Based on Scanning Electron Microscope" was retracted in 2023. Reasons: unreliable results or conclusions; concerns about the data; concerns about the peer review; concerns about the citations.

### 3.6. Effect of Fermentation Days on Bacterial Cellulose Fermentation

The shaking time of carbon source glucose seed solution in fermentation medium used by three strains of Acetobacter xylobacter was selected for 30 hours, and then, 50 mL of carbon source glucose seed solution was inoculated into fermentation medium at an inoculation rate of 8% and incubated for 10 days at a constant temperature starting at 5 and 30, respectively. Samples were taken every two days to measure the change in yield and the concentration of residual carbon source in fermentation liquid. The carbon source utilization rate and cellulose conversion rate of the three strains were calculated [21].

(1) $$\begin{array}{c} \text{Carbon source utilization ratio }\left(\%\right)=\left(\text{initial carbon source concentration}-\text{final carbon source concentration}\right)\text{or initial carbon source concentration},\\ \text{BC percent conversion }\left(\text{g}/\text{g}\right)=\frac{\text{BC output}}{\text{Total initial carbon source}-\text{Total final carbon source}}. \end{array}$$

### 3.7. Determination of Residual Sugar in Fermentation Broth

The DNS method was used to prepare standard glucose solution; then, 10 test tubes (25 mL) were taken, and corresponding reagents were added according to Table 5. Then, DNS reagents were added, respectively, and the boiling water bath was conducted for 5 minutes.  Figure 2 shows the blood glucose standard curve. After cooling, deionized water was added. After mixing, the absorption value was measured at the wavelength with the standard glucose concentration as the abscissa and the absorbance value as the ordinate. The standard curve was drawn, and the regression equation was calculated [22].

### 3.8. Observing Colloidal Structure

BC/PVA/PEG composite hydrogel: add corresponding PEG to the dissolved PVA solution, place it in a water bath, and form a homogeneous solution after mixing. After mechanical dewatering, the thickness of the purified membrane was about, and the membrane was immersed in the corresponding mixed solution of PVA and PEG. The impregnation and freeze-thaw process were the same as above, and the freeze-thaw process was repeated for 2-6 times to obtain the composite BC/PVA/PEG hydrogel [23].

The article "Preparation and Performance Analysis of Bacterial Cellulose-Based Composite Hydrogel Based on Scanning Electron Microscope" was retracted in 2023. Reasons: unreliable results or conclusions; concerns about the data; concerns about the peer review; concerns about the citations.

The prepared bacterial cellulose film was freeze-dried and sprayed with gold; then, the microspatial structure and colloid mesh aperture of bacterial cellulose were observed by BSE SEI scanning electron microscope, and the micromorphology of BC and its composite hydrogels were observed by scanning electron microscope [24].

## 4. Results and Discussion

Experiments show that the three-dimensional network observed by scanning electron microscope has a dense structure with criss-crossing fibers and an average size of 40-60 nm. The corresponding results are as follows: the gel preparation effect is the most ideal when PEG concentration is below 6%. In addition, adding the following PEG will not produce a significant increase in hydrophobicity of phase separation when PEG concentration is above [25].

## 5. Conclusion

This paper presents an experimental method based on scanning electron microscope. The specific content of this method is to observe the hydrogel through scanning electron microscope and observe the intermolecular space through experiment to prove the effect of this method to solve the problem of preparing hydrogel from bacterial cellulose. Bacterial cellulose is a kind of biocellulose with high application value. It has many excellent physical and chemical properties. However, in practical application, some properties of bacterial cellulose cannot meet the requirements perfectly, so its structural characteristics need to be improved.

## Figures and Tables

**Figure 1:** Preparation of collagen-based hydrogel.

**Figure 2:** Glucose standard curve.

**Table 1:** Characteristics of bacterial cellulose species.

Bacterial genus	Cellulose characteristics	Crystal form	Function
Acetobacter	Extracellular membrane cellulose	Type I of type II	Aerobic environment
Rhizobium	Extracellular microfibers	Type I	Adsorb to parasitic plants
Agrobacterium	Extracellular microfibers	Type I	Adsorb to plant tissue
Sarcina	Amorphous cellulose	Type I	Unclear

**Table 2:** Test reagent list.

Name	Molecular formula	Actual size
Glucose	C_6_H_12_O_6_	Analytically pure
Xylose	C_5_H_10_O_5_	Analytically pure
Galactose	C_6_H_12_O_6_	Analytically pure
Arabinose	C_5_H_10_O_5_	Analytically pure
Mannose	C_12_H_22_O_11_	Analytically pure
Tryptone		Biochemical reagent
Yeast		Biochemical reagent
Citric acid	C_6_H_8_O_7_·H_2_O	Analytically pure
Agar powder		Biochemical reagent
3,5-Trinitro	C_7_H_4_N_2_O_7_	Analytically pure
Trinitro-seignette salt	C_4_H_4_KNaO_6_·_4_H_2_O	Analytically pure
Phenol	C_6_H_5_OH	Analytically pure
Anhydrous sodium sulfate	Na_2_SO_4_	Analytically pure
Sodium hydroxide	NaOH	Analytically pure

**Table 3:** Experimental apparatus.

Name of instrument	Model
Sartorius electronic scales	BS224
Magnetic stirring apparatus	85-1B
Lightning magnetic laboratory digital pH meter	PHSJ-4A
Automatic autoclave cooker	YXQ-LS-SH
Peying full temperature control shaker	HYG-B
Water-jacket incubator	9080
Double single clean table	SW-CJ-2FD
Digital display electric thermostatic water bath	XMTB
Electrothermostatic blast oven	DHG-914OA
Lyophilizer	Alpha 1-2 LD
Scanning electron microscope	BSESEI
Fully automatic specific surface and porosity analyzer	TriStar II 3020
Fourier transform infrared Raman spectroscopy	NEXUS-670

The article "Preparation and Performance Analysis of Bacterial Cellulose-Based Composite Hydrogel Based on Scanning Electron Microscope" was retracted in 2023. Reasons: unreliable results or conclusions; concerns about the data; concerns about the peer review; concerns about the citations.

**Table 4:** Orthogonal experimental factors and level tables.

	Bacterial strain	Inoculum age	Inoculum size
1	ATCC23770	18 h	6%
2	ZGD201301	24 h	8%
3	ATCCZ200801	30 h	10%

**Table 5:** DNS sample list.

Glucose (mL)	0.1	0.2	0.3	0.4	0.5	0.6	0.7	0.8	0.9	1.0
Water (mL)	0.9	0.8	0.7	0.6	0.5	0.4	0.3	0.2	0.1	0
Sugar concentration (mg/mL)	0.2	0.4	0.6	0.8	1.0	1.2	1.4	1.6	1.8	2.0

## Data Availability

The data used to support the findings of this study are available from the corresponding author upon request.
